The article "Magnetic Resonance Image Compilation Was Used in Conjunction with Prostate PI-RADS v2.1 Score Has Diagnostic Relevance for Benign and Malignant Prostate Lesions" was retracted in 2023. Reasons: unreliable results or conclusions; concerns about the data; concerns about the peer review; concerns about the citations.

# Magnetic Resonance Image Compilation Was Used in Conjunction with Prostate PI-RADS v2.1 Score Has Diagnostic Relevance for Benign and Malignant Prostate Lesions

**DOI:** 10.1155/2022/3613540

**Published:** 2022-08-29

**Authors:** Wenjuan Xu, HaiYan Cao, Fang Du, Ling He, FangLian Jiang, ChunHong Hu

**Affiliations:** ^1^Department of Radiology, The First Affiliated Hospital of Soochow University, Suzhou, Jiangsu Province 215006, China; ^2^Department of Radiology, Medical Image Center, The Affiliated Hospital of Yangzhou University, Yangzhou, Jiangsu Province 225001, China; ^3^Department of Ultrasound, Yancheng First Hospital, Affiliated Hospital of Nanjing University Medical School(the First People, S Hospital of Yancheng), Yancheng, Jiangsu Province224001, China

## Abstract

**Objective:**

To assess the diagnostic usefulness of magic in conjunction with PI-RADS v2.1 for prostate cancer malignant foci.

**Methods:**

A total of 202 lesions (97 transitional zone lesions and 105 peripheral zone lesions) from 198 people were investigated retrospectively using traditional MRI and magic images. Each lesion has a unique pathological consequence. Lesions T1, T2, and PD values were employed as magic observation markers. The locations of the lesions were aggregated, and the paired *t*-test and receiver operating characteristic curve (ROC) were employed to find the indices with statistical significance in separating benign from malignant prostatic nodules (+1 point) and (−1 point) respectively. Draw a ROC curve and compare it to the PI-RADS v2.1 score using the magic positive and negative indices as well as the PI-RADS v2.1 score. By comparing the ROC curves scored separately, the diagnostic efficiency of the two scoring approaches for benign and malignant prostate lesions was investigated.

**Results:**

T2 value has the highest diagnostic efficiency among the magic observation indices. T2 value of 77 ms for transitional zone lesions and T2 value of 89 ms for peripheral zone lesions are positive indices, whereas T2 value >77 ms and T2 value >89 ms are negative indexes. PI-RADS v2.1 combines one score and magic. In the transitional zone, the sensitivity, specificity, positive predictive value, and negative predictive value of the two scoring methods were 57.52, 87.70, 76.70, and 74.6 percent and 82.50, 73.68, 95.5, and 74.7 percent, respectively, and the AUC values were 0.735 and 0.846, respectively (*P* = 0.004); in the peripheral zone, the AUC values were 86.15 percent, 68.42 percent, 82.4.

**Conclusions:**

Magic T2 value is a favorable sign for diagnosing benign and malignant prostate cancers when used in conjunction with PI-RADS v2.1. The end product exceeds PI-RADS v2.1 on its own, which is more useful in identifying benign and malignant prostate lesions, decreasing unnecessary puncture and alleviating patient pain.

The article "Magnetic Resonance Image Compilation Was Used in Conjunction with Prostate PI-RADS v2.1 Score Has Diagnostic Relevance for Benign and Malignant Prostate Lesions" was retracted in 2023. Reasons: unreliable results or conclusions; concerns about the data; concerns about the peer review; concerns about the citations.

## 1. Introduction

Prostate cancer (PCA) is the world's second most frequent male cancer and the fourth major cause of cancer mortality in males [1, 2]. Early detection and appropriate staging seem to be particularly critical for PCA therapy and prognosis [3]. Digital rectal examination, traditional transrectal ultrasound (TRUS)-guided biopsy, PSA testing, and magnetic resonance imaging are now used to diagnose prostate disease (MRI). MRI, with its excellent soft tissue contrast capacity and noninvasive nature, has been extensively employed in the identification, localization, and staging of benign and malignant prostate tumors [2]. The first and second editions of the prostate imaging reporting and data system (PIRADS) were introduced, respectively, at the 2012 annual European Urogenital Radiology meeting, the 2014 American College of Radiology, and the European Society of Urogenital Radiology joint AdMeTech foundation, to standardize MRI image acquisition, image interpretation, and report writing, as well as to improve diagnostic accuracy and reduce unnecessary punctures for benign and malignant prostate. In 2019, this data system was upgraded to PI-RADS v2.0 Version 1 of the PI-RADS data system application streamlines reporting and scanning definitions, as well as surgeon and patient interpretation of findings. Previous clinical investigations have also shown that the PI-RADS score system correlates better with clinical diagnoses [4].

These quantitative approaches, such as apparent diffusion coefficient (ADC), diffusion kurtosis imaging (DKI), diffusion tensor imaging (DTI), and intravoxel incoherent motion (IVIM), have been increasingly employed for MRI detection of prostate disorders in recent years [5, 6]. Magic (magnetic resonance image preparation), also known as synthetic MRI, has recently developed a new MRI quantitative sequence, one-stop relaxation quantitative MRI, by optimizing the multi delay versus multi echo technique with saturation pulses alternating with signal acquisition and additionally incorporating estimation and correction for radiofrequency field inhomogeneities. The relaxation periods and proton density were quantified using a multisaturation recovery multiecho paired fast spin echo readout. Its benefit is its capacity to give absolute quantitative maps of T1, T2, and PD maps in a single scan, giving objective quantitative data for illness diagnosis. The purpose of this research was to look into the cutoff values of magic technology in distinguishing benign from malignant prostate disorders, as well as the combination of magic-related quantitative factors with prostate PI-RADS v2.1 score value for the correction of benign and malignant prostate lesions.

The article "Magnetic Resonance Image Compilation Was Used in Conjunction with Prostate PI-RADS v2.1 Score Has Diagnostic Relevance for Benign and Malignant Prostate Lesions" was retracted in 2023. Reasons: unreliable results or conclusions; concerns about the data; concerns about the peer review; concerns about the citations.

## 2. Materials and Methods

### 2.1. Study Subjects

Patients with routine pathology findings who had prostate puncture or surgery in our institution between October 2020 and December 2021 had their MR imaging data evaluated retrospectively. Inclusion criteria are as follows: (1) no medication or surgical therapy prior to prostate MRI examination; (2) no needle biopsy performed prior to the prostate MRI test; and (3) all patients receiving the magic examination. Exclusion criteria are as follows: (1) no pathological findings after magnetic resonance examination and a time interval of more than 3 months between biopsy and MRI examination; (2) lesions in the context of diffuse type lesions of the prostate; (3) prostate lesions ≤5 mm; (4) insufficient data on MRI imaging; and (5) magnetic resonance images of poor quality with significant image artifacts. This study included 198 patients, 202 lesions, 97 of which were transitional band lesions and 105 of which were peripheral band lesions, with the most common complaints being PSA elevation or/and urinary frequency, dysuria, urinary retention, hematuria, and other symptoms; radical prostatectomy was performed in 129 patients (58 lesions in the peripheral band and 71 lesions in the transitional band). The medical ethics review board of Yangzhou University's Affiliated Hospital authorized this research, and all patients provided written informed permission. The age range was 29-87 years old, with a mean age of (68.48 ±0.69)

### 2.2. MRI Scanning Techniques

The scanner utilized was a GE- architect 3.0 T MRI scanner with 16 channel coils (anterior array, AA) and a 40 channel coil (posterior array). Before the examination, the patient's urine was correctly preserved, and the scan body position comprised axial, coronal, and sagittal, with the axial direction perpendicular to the long axis of the prostate. T1WI and T2WI scans with rapid spin echo sequences, small field high-resolution T2WI and DWI scans, DCE scans (DCE scans were not frequently conducted), and magic scans were among the sequences used. Axial parameters for T1WI sequences were entered: repetition time (TR) =620 ms, echo time (echo time, TE) =15 ms, slice thickness/interslice spacing 3.0 mm/0 mm, scan field 200×200 mm, matrix (matrix) 320×320, number of excitations (nex) 2 times, and image duration 2 min 35 s. On T1WI sequences, the following parameters were used: TR =620 ms, TE= 15 ms, slice thickness/interslice distance 3.0 mm/0 mm, scan field 340×340 mm, matrix 320×320, nex 2 times, and picture duration 2 minutes 28 seconds. On T2WI sequences, the axial parameters were TR =3500 ms, TE =100 ms, slice thickness/interslice distance 3.0 mm/0 mm, scan field 200 ×200 mm, matrix 320×320, nex 2.5 times, and picture duration 2 minutes 28 seconds. On T2WI sequences, the coronary parameters were TR =3700 ms, TE =106 ms, slice thickness/interslice distance 3.0 mm/0 mm, scan field 340 ×340 mm, matrix 320×320, nex 2.5 times, and image duration 2 minutes 14 seconds. On T2WI sequences, the sagittal parameters were TR = 4100 ms, TE = 140 ms, slice thickness /interslice distance = 3.0 mm / 0 mm, scan field = 280×280 mm, matrix 320×320, nex 2 times,and picture acquisition duration 2 minutes 6 seconds. On DWI sequences, the axialparameters were TR=3600 ms,TE=86 ms, slice thickness / interslice distance 3.0mm / 1.0 mm, scan field 280×140 mm, matrix 120× 60, nex 2 times, picture duration 2 minutes 6 seconds.On MAGIC sequencws, the axial parameters were TR= 4300ms, TE= 20 / 108ms, slice thickness/ slice spacing 3.0mm/0.5mm, scan field of view 300×300 mm, matrix 320×256, nex 1 time,picture time 4 minutes 23 seconds.On DCE sequencesTR= 5 ms, TE = 2 ms, slice thickness / interslice distance 6.0 mm / 0 mm, scan field = 288 ×245 mm, matrix 224×192, no nex, picture collection time 5min 6 s, total scan duration 30 periods.The time resolution is 10 seconds. tr = 4100 MS, TE = 140 ms, slice thickness/interslice distance = 3.0 mm/0 mm, scan field = 280 280 mm, Gadopentetate dimeglumine (GD DTPA) was given intravenously by the elbow using a two barrel high-pressure syringe at an injection rate of 2–3 ml/s and a bolus of 0.1 mmol/kg in 20 ml tubes.

The article "Magnetic Resonance Image Compilation Was Used in Conjunction with Prostate PI-RADS v2.1 Score Has Diagnostic Relevance for Benign and Malignant Prostate Lesions" was retracted in 2023. Reasons: unreliable results or conclusions; concerns about the data; concerns about the peer review; concerns about the citations.

### 2.3. Pathological Examination and Zonation

Rectal ultrasonography was used to identify the perineal route after MRI in 198 patients, and the puncture was performed by an experienced chief physician who preoperatively analyzed the patient's MRI data and coordinated with the imaging physician to determine the targeted puncture. Ultrasonography-magnetic resonance fusion navigation biopsy (TRUS-MRI FB) and ultrasound-guided systematic biopsy (TRUS-SB) “10 needles” combined prostate puncture method TRUS and guided the piercing of the MRI-targeted targets. TRUS-MRI fusion navigation puncture (TRUS-MRI FB) and ultrasound-guided system puncture (TRUS-SB) prostate puncture method TRUS guided the piercing of the MRI-targeted targets. Each chosen target received 2-4 needles; conventional puncture used 10 needles, one for each of the prostate's peripheral bands, notably the anterior, lateral, central, paramedian, and transitional bands (Figure 1). In this research, histopathological samples of radical prostatectomy were chosen as the ultimate pathological reference for individuals who had simultaneous radical prostatectomy and biopsy.

The article "Magnetic Resonance Image Compilation Was Used in Conjunction with Prostate PI-RADS v2.1 Score Has Diagnostic Relevance for Benign and Malignant Prostate Lesions" was retracted in 2023. Reasons: unreliable results or conclusions; concerns about the data; concerns about the peer review; concerns about the citations.

### 2.4. Image Processing and PI-RADS v2.1 Scoring Criteria

The scanned images were sent to a diagnostic workstation, and the enrolled cases were co-analyzed in a double blinded manner by two physicians with more than 5 and 10 years of experience in MRI diagnosis and analyzed according to find PI-RADS v2.1 standard scoring, with consensus achieved when scoring was discordant [7, 8]. The peripheral zone of the prostate (PZ) is dominated by DWI (ADC) scores, such as: DWI (ADC) of 3 points, T2WI is arbitrary, DCE is negative, and the total score remains unchanged, remaining 3 points; DCE was positive with a total score of 3 +1, which was 4 points. T2WI scores dominated the transitional zone (TZ), for example: T2WI of 2 points, if DWI (ADC) ≤ 3 points, total score unaltered, if DWI (ADC) ≥ 4 points, and total score 3 points; T2WI of 3 points, DWI (ADC) ≤ 4 points, total score unaltered, if DWI (ADC) of 5 points, total score 4 points, and negative or positive DCE in the mobility band score had no effect on the overall score. Finally, use the PI-RADS v2.1 score to determine the probability of PCA: 1 point = very unlikely to exist; 2 points = unlikely to be present; 3 points = dubious existence; 4 points = probable presence; and 5 points = highly likely to be present. In our research, the biggest diameter of the lesion was at the PZ according to the PZ score, and the largest diameter was at the TZ according to the TZ score of the migrating band, when the lesion was substantial and included either the PZ or the TZ. Two radiologists (with over 5 and 10 years of experience in MRI diagnostic work-up, respectively) manually drew the area of interest (ROI) based on T2WI and DWI images based on the pathological findings. For each enrolled case, GE aw4 was used to create a ready view in the system. First, the prostate tissue was mirror segmented, and two levels displaying the most typical clarity of prostate cancer were chosen to avoid necrosis, cystic change, hemorrhage areas, and so on, and the dedicated magic postprocessing software on the GE- architect device was used to acquire T1 value, T2 value, and PD value of the focal area of the prostate (Figure 2).

### 2.5. Statistical Methods

Results were analyzed using SPSS21.0 statistical software, and measurement data were represented as mean standard deviation (x ± s). The intergroup comparison of counting data was done using paired *t*-test to establish the differential indicators of the magic approach in discriminating benign and malignant prostate cancers, and *P* < 0.05 was judged statistically significant. If there was more than one statistically significant indication, the differential indicators were scored again (1 point for the positive indicator and −1 point for the negative indicator). Using the MedCalc 19.2 statistical program, the differential index of the final inclusion score was derived by calculating the receiver operating characteristic curve (ROC) and comparing the area under the curve with pathological results as status factors (AUC). PI-RADS v2.1 was plotted separately with pathological findings as the status variable scoring, the *Z*-test was used to compare the difference between the AUCs, and the MAGIC combined PI-RADS v2.1 ROC curve of the score was used to determine its optimal diagnostic cut-off value, sensitivity, specificity, positive predictive value (PPV), and negative predictive value (NPV) in the diagnosis of benign and malignant lesions of the prostate.

The article "Magnetic Resonance Image Compilation Was Used in Conjunction with Prostate PI-RADS v2.1 Score Has Diagnostic Relevance for Benign and Malignant Prostate Lesions" was retracted in 2023. Reasons: unreliable results or conclusions; concerns about the data; concerns about the peer review; concerns about the citations.

## 3. Results

### 3.1. Pathological Findings

In the peripheral band region, all 202 lesions from 197 individuals displayed unambiguous conventional pathology findings, including 40 (38.1%) benign and 65 (61.9%) malignant lesions. The benign nodules had a maximum diameter of 5-24 mm and a mean diameter of 11.8-64.77%; the malignant nodules had a maximum diameter of 5-27 mm and a mean diameter of (13.1-95.19%). In the group of peripheral benign and malignant lesions, the transitional zone was home to 57 (58.78%) benign lesions and 40 (41.2%) malignant lesions. The benign nodules had a maximum diameter of 7-38 mm and a mean diameter of 13.93 ± 6.17 mm; the malignant nodules had a maximum diameter of 3-30 mm and a mean diameter of 15.82 ± 6.87 mm.

### 3.2. PI-RADS v2.1 Ratio of Benign to Malignant Lesion Composition in Different Scores

The prostatic lesions included in this investigation had PI-RADS values of 2, 3, 4, and 5. The percentage of malignant foci with shifted bands in PI-RADS 2-5 scores was 0.25%, 76%, 75.22%, and 83.33%; the percentage of peripheral band malignant foci in PI-RADS 2-5 scores was 0%.31.03%, 74.51%, and 94.74% (see Table 1).

#### 3.2.1. Differences in Quantitative Parameters of Benign and Malignant Lesions of the Prostate

Table 2 shows the T1, T2, and PD values in benign and malignant prostate tumors. T1, T2, and PD values were lower in transitional and peripheral PCA lesions than in noncancerous regions. T1 and T2 values of PCA lesions in the transitional zone were lower than those of benign hyperplasia (*P* = 0.03, 0.001), and PD values of PCA lesions were not significantly different from those of benign hyperplasia (*P* = 0.209); T2 value was significantly different (*P* < 0.001) between peripheral band PCA and non cancerous tissue, while T1 and PD values were not significantly different (*P* = 018, 0.25).

The article "Magnetic Resonance Image Compilation Was Used in Conjunction with Prostate PI-RADS v2.1 Score Has Diagnostic Relevance for Benign and Malignant Prostate Lesions" was retracted in 2023. Reasons: unreliable results or conclusions; concerns about the data; concerns about the peer review; concerns about the citations.

#### 3.2.2. Diagnostic Efficacy of Different Quantitative Parameters in Differentiating Benign and Malignant Foci of Prostate

Figure 3 depicts the findings of ROC analysis of the quantitative parameters T1, T2, and PD values of the migrating and peripheral bands in distinguishing benign from malignant tumors. The AUC of T2 value was significantly higher than that of T1 and Pd (*P* = 0.0063 and 0.0023, respectively) for discriminating PCA from benign hyperplasia in the region of the migrating band, and the AUC of T1 value was slightly higher than that of PD value without statistical significance (*P* = 0.3683). For PCA and noncancerous tissue discriminating peripheral band regions, the AUC of T2 value was still significantly higher than that of T1 and Pd (the AUC values of T2 value in the migrating band and peripheral band sections in this research were 0.819 and 0.813, respectively).

### 3.3. PI-RADS v2.1 Scoring and T2 Values Combined PI-RADS v2.1 Diagnostic Efficacy for Benign and Malignant Lesions of the Prostate

T2 values in this research demonstrated good diagnostic effectiveness in the identification of benign and malignant prostate disorders, with cutoffs of 77 ms for T2 values in the transitional zone and 89 ms for T2 values in the peripheral zone. The sensitivity, specificity, PPV, and NPV of the two scoring methods, PI-RADS V2.1 scoring and T2 value, combined with PI-RADS V2.1 scoring in the diagnosis of benign and malignant diseases of the prostate transitional zone were 57.52, 87.70, 76.70, and 74.6 percent and 82.50, 73.68, 95.5, and 74.7 percent, respectively, and the AUC values were 0.735 and 0.846, respectively (see Table 3). The sensitivity, specificity, PPV, and NP are shown in Table 4. The combination of PI-RADS v2.1 scores and quantitative parametric T2 value demonstrated a higher diagnostic value for benign and malignant prostate lesions, regardless of whether they were migration band or peripheral band lesions (migration band *z* = 2.878, *P* = 0.0040; peripheral band *z* = 2.103, *P* = 0.0355), as shown in Figure 4.

## 4. Discussion

PI-RADS, a standardized reporting system for magnetic resonance diagnostic of prostate imaging, was released in 2012 by the European Society of Urological Radiology (ESUR). The American College of Radiology, the European Society of Genitourinary Radiology, and the AdMeTech Foundation scoring standards released PI-RADS v2.0 in September 2015, with improved diagnostic expertise and scanning methodology. Previous study has demonstrated that the PI-RADS v2.0 scoring system is useful for diagnosing prostate cancer and increases the positive rate of prostate puncture. [9]. The most current prostate magnetic resonance scoring version PI-RADS v2.1, proposed in 2019 by European Urology, is more granular and selective, decreasing PI-RADS v2.0 The existence of confusing scoring standards, as well as a lack of definition of scoring zones, improves the diagnostic consistency and accuracy of prostate cancer [10]. Nonetheless, owing to the absence of a specific value of objective quantitative parameters, the interobserver agreement might still have some impact due to the expertise level of various readers, often resulting to larger false-positive findings and limiting the detection rate of PCA [11].

The article "Magnetic Resonance Image Compilation Was Used in Conjunction with Prostate PI-RADS v2.1 Score Has Diagnostic Relevance for Benign and Malignant Prostate Lesions" was retracted in 2023. Reasons: unreliable results or conclusions; concerns about the data; concerns about the peer review; concerns about the citations.

Magic (magnetic resonance image preparation), also known as synthetic MRI, is a ground-breaking one-stop relaxation quantitative MR method capable of detecting T1, T2, and PD values in a single scan. Originally, Magic was intended for use in imaging the central nervous system [12] and then gradually expanded into other systems, primarily on organs with less respiratory activity. It was originally intended for use in imaging the central nervous system and gradually expanded into other systems, primarily in organs with less respiratory activity. There has been little study on its application to prostate illness; however, Cui Yadong et al. investigated the use of quantitative parameters produced from synthetic MR imaging technology for the detection of prostate cancer [13]. However, since the importance of quantitative parameters T1, T2, and PD values in the diagnosis of prostate disease is not widely accepted, this approach was not included in its scoring system. In this study, we looked for the most meaningful quantitative parameter values for the diagnosis of prostate cancer by interpreting and statistically analyzing different quantitative parameters (T1, T2, and PD values) between prostate cancer and noncancerous areas, and we determined the possible positive and negative indicators for the diagnosis of prostate cancer, counting +1 point for the positive indicator and − 1 point for the negative indicator, and we went on to investigate further. Also, talk about if its diagnostic accuracy has increased.

The nodules in this study were all PI-RADS scores 2-5, and the percentage of peripheral band prostate cancer in PI-RADS 2-5 points was 0.31.03, 74.51, and 94.74 percent, and the percentage of transitional band malignant lesions in PI-RADS 2-5 points was 0.25.76, 75.22, and 83.33 percent, which was similar to PI-RADS v2.1 score guideline's accompanying risk of malignancy was fulfilled. The individuals in this investigation with PI-RADS 2-points lesions all exhibited elevated blood prostate-specific antigen levels (> 10 ng/ml) (PSA). We scored 202 lesions by PI-RADS scoreing and generated ROC curves for the quantitative parameters T1, T2, and PD values, respectively, and determined that the quantitative parameter values with the most diagnostic efficacy for prostate cancer were T2 value, shifted band diagnostic value was 77 ms, and peripheral band diagnostic value was 89 ms, which was generally consistent with measurements in previous studies [13, 14].

The article "Magnetic Resonance Image Compilation Was Used in Conjunction with Prostate PI-RADS v2.1 Score Has Diagnostic Relevance for Benign and Malignant Prostate Lesions" was retracted in 2023. Reasons: unreliable results or conclusions; concerns about the data; concerns about the peer review; concerns about the citations.

In this work, we looked at 202 lesions to determine the utility of the magic quantitative parameter maps T1, T2, and PD values in distinguishing PCA lesions from other benign tumors. The T2 values of the lesions were highly significantly different between benign and malignant lesions (*P* = 0.001), the T1 values were statistically different between benign and malignant lesions (*P* = 0.03 for the shifted band and *P* = 0.018 for the peripheral band), and the PD values, although the differences between benign and malignant lesions were not statistically significant for the shifted band (*P* = 0.209), The majority of prior investigations focused on peripheral band prostate cancer and discovered that PCA lesions had considerably lower T2 values than normal PZ [15–17]. The present study's results are consistent with previous studies in that T2 levels are critical in differentiating PCA from non-neoplastic PZ lesions in peripheral bands. Some studies found no statistically significant difference in T2 values between PCA lesions with misplaced bands and hyperplastic prostatic nodules (BPH) [18]. However, one investigation found that transitional PCA lesions had lower T2 values than nontumor TZ lesions [19]. The current research also discovered that T2 values in the transitional band of PCA lesions were considerably lower than those in non-cancerous tissue.

We also discovered that T2 values of transitional band and peripheral band lesions were substantially more efficient than T1 and PD values in distinguishing benign and cancerous prostate. T1 value exhibited slightly greater diagnostic effectiveness than PD value for prostate cancer lesions with a transitional band, but there was no statistical significance between them (*P* = 0.3683); for peripheral band lesions, T1 value had almost the same diagnostic efficiency as PD value. In this investigation, the AUC of the T2 value in distinguishing peripheral band PCA lesions from non-tumor PZ lesions was 0.813, which was comparable to the findings of a previous study [20]. The AUC of T2 value was 0.819 for the discriminating of PCA lesions and benign hyperplasia in the transitional zone, and the diagnostic effectiveness was greater than that of T1 and PD values, and the findings of earlier investigations (AUC 0.840) were nearly comparable [21]. Because T2 value has been recognized as a quantitative marker reflecting free water in tissues, in prostate cancer patients, the normal free water inside the loose interstitium between the ducts and acini is replaced by densely packed malignant epithelial cells, the free water in the extracellular space is significantly reduced, and thus the T2 value is significantly reduced [22]. Despite being an intrinsic property quantitative parameter of the tissue itself, T1 and PD values were shown to be less effective than T2 value in the research and hence were not deemed positive indications.

The article "Magnetic Resonance Image Compilation Was Used in Conjunction with Prostate PI-RADS v2.1 Score Has Diagnostic Relevance for Benign and Malignant Prostate Lesions" was retracted in 2023. Reasons: unreliable results or conclusions; concerns about the data; concerns about the peer review; concerns about the citations.

In this study, we discovered that T2 value combined with PI-RADS v2.1 score was more valuable than PI-RADS v2.1 alone in the diagnosis of prostate cancer, with AUC values of 0.735 and 0.846 for the shifted band and 0.816 and 0.890 for the peripheral band, which were significantly different (*P* = 0.0355), and the 95 percent confidence intervals of the shifted band versus peripheral band, which were significantly different (*P* = 0.0355), and when compared to the PI-RADS v2.1 score, T2 value coupled with PI-RADS v2.1 score not only showed higher diagnostic efficacy in the diagnosis of benign and malignant prostate, but also had more trustworthy diagnostic results [23]. The current study's findings show that the main improvements in the T2 value combined with the PI-RADS v2.1 score over the PI-RADS v2.1 score in the diagnosis of benign and malignant prostate transitional zone lesions are diagnostic sensitivity and positive predictive value; the main improvements in the diagnosis of benign and malignant prostate peripheral zone lesions were specificity and positive predictive value, demonstrating that the combined score can effectively detect lesions. As a result, the authors propose that lesions with shifting band T2 value >77 ms and peripheral band T2 value >89 ms may be followed up on without needless prostate ultrasound-guided puncture to alleviate patient suffering. Shifting band T2 value 77 ms, peripheral band T2 value 89 ms, or more lesions imply the necessity for prostate ultrasound-guided targeted puncture to increase the diagnostic yield of puncture. The current research contains significant flaws. First and foremost, this is a retrospective research with the potential for bias in patient selection, which requires multicenter or prospective trials to confirm. Second, some of the pathology results in this research were from prostate needle biopsies, which raise the chance of prostate cancer being overlooked. The current research is novel in that it is now vital to combine PI-RADS v2.1 for T2 value in prostate illness, which has received little attention.

The article "Magnetic Resonance Image Compilation Was Used in Conjunction with Prostate PI-RADS v2.1 Score Has Diagnostic Relevance for Benign and Malignant Prostate Lesions" was retracted in 2023. Reasons: unreliable results or conclusions; concerns about the data; concerns about the peer review; concerns about the citations.

## 5. Conclusion

In conclusion, PI-RADS v2.1 score, when paired with the magic quantitative parameters, demonstrated great diagnostic effectiveness for the detection of prostate cancer using T2 value mixed with PI-RADS v2.1.

## Figures and Tables

**Figure 1:** Prostate sb 10 gauge. The puncture points of (a)–(j) were the following: anteroposterior, lateral, medial, and paramedian of the right peripheral band and the paramedian, medial, lateral, and anteroposterior of the left peripheral band and the transitional band on the right side; (k)–(l) is the pathology result of puncture; immunohistochemistry results are prostate hyperplasia.

**Figure 2:** Migrated magic images with prostate cancer. (a) is the T2WI, (b) is the T1 value, (c) is the T2 value, (d) is the PD value, (e) is the small field T2W fat pressing axial, (f) is the diffusion-weighted image with *b* value 2000, and (g) is the pathological result of prostate cancer.

**Figure 3:** ROC curves showing the diagnostic efficacy of T1, T2, and PD values in the migration band and peripheral band areas for differentiating benign and malignant lesions of prostate.

**Figure 4:** ROC curves of the diagnostic values of the two scoring methods for benign and malignant lesions of the prostate.

**Table 1:** PI-RADS scores and the ratio of benign to malignant composition of prostate lesions on MP MRI.

PI-RADS score	Transitional zone		Total	Malignant rate	Peripheral zone		Total	Malignant rate
	Benign	Malignant			Benign	Malignant		
2	1	0	1	0%	6	0	6	0
3	49	17	66	25.76%	20	9	29	31.03%
4	5	13	18	72.22%	13	38	51	74.51%
5	2	10	12	83.33%	1	18	19	94.74%

**Table 2:** results of different quantitative parameters for benign and malignant lesions of prostate.

TumoR character	Transitional zone			Peripheral zone		
	T1 (ms)	T2 (ms)	PD (pu)	T1 (ms)	T2 (ms)	PD (pu)
Benign proliferation/noncancerous tissue	1561.72 ± 326.08	99.98 ± 13.51	71.80 ± 7.77	2003.27 ± 480.33	132.63 ± 39.50	76.73 ± 8.74
Prostatic	1228.92 ± 302.30	80.04 ± 11.63	67.53 ± 8.33	1310.13 ± 237.64	86.03 ± 14.16	68.87 ± 6.78
*t*	3.037	5.859	-1.386	2.412	5.787	2.280
*p*	0.03	<0.001	0.209	0.018	<0.001	0.025

**Table 3:** Comparison of the two scoring methods for the diagnosis of benign and malignant transitional zone lesions.

Scoring method	Susceptibility (%)	Specificity (%)	PPV (%)	NPV (%)	AUC	95% CI
PI-RADS v2.1	57.52	87.70	76.7	74.6	0.735	0.636~ 0.820
PI-RADS v2.1 + T2	82.5	73.68	95.5	74.7	0.846	0.759~ 0.911

**Table 4:** Comparison of the diagnostic values of the two scoring methods for benign and malignant peripheral band lesions peripherin.

Scoring method	Susceptibility (%)	Specificity (%)	PPV (%)	NPV (%)	AUC	95% CI
PI-RADS v2.1	86.15	68.42	82.4	74.3	0.816	0.728~ 0.886
PI-RADS v2.1 + T2	70.8	92.1	93.9	64.8	0.890	0.813~ 0.943

The article "Magnetic Resonance Image Compilation Was Used in Conjunction with Prostate PI-RADS v2.1 Score Has Diagnostic Relevance for Benign and Malignant Prostate Lesions" was retracted in 2023. Reasons: unreliable results or conclusions; concerns about the data; concerns about the peer review; concerns about the citations.

## Data Availability

All of the data in this article is actually available.

## References

[1] Bray F., Ferlay J., Soerjomataram I., Siegel R. L., Torre L. A., Jemal A. (2018). Global cancer statistics 2018: GLOBOCAN estimates of incidence and mortality worldwide for 36 cancers in 185 countries. *CA: a Cancer Journal for Clinicians*.

[2] Gong X., Wu K., Hao S. (2019). A comparative study on the diagnostic value of MRI dynamic enhancement in prostate cancer reporting and data systems 1.0 and 2.0. *Chinese Journal of Medical Computer Imaging*.

[3] Turkbey B., Rosenkrantz A. B., Haider M. A. (2019). Prostate imaging reporting and data system version 2.1: 2019 update of prostate imaging reporting and data system version 2. *European Urology*.

[4] Park S. Y., Jung D. C., Oh Y. T. (2016). Prostate cancer: PI-RADS version 2 helps preoperatively predict clinically significant cancers. *Radiology*.

[5] Wang X., Tu N., Qin T., Xing F., Wang P., Wu G. (2018). Diffusion kurtosis imaging combined with dwi at 3-t mri for detection and assessment of aggressiveness of prostate cancer. *AJR. American Journal of Roentgenology*.

[6] Pavilla A., Gambarota G., Arrigo A., Mejdoubi M., Duvauferrier R., Saint-Jalmes H. (2017). Diffusional kurtosis imaging (DKI) incorporation into an intravoxel incoherent motion (IVIM) MR model to measure cerebral hypoperfusion induced by hyperventilation challenge in healthy subjects. *Magma*.

[7] Liu C., Liu S. L., Wang Z. X. (2018). Using the prostate imaging reporting and data system version 2 (PI-RIDS v2) to detect prostate cancer can prevent unnecessary biopsies and invasive treatment. *Asian Journal of Andrology*.

[8] Byun J., Park K. J., Kim M. H., Kim J. K. (2020). direct comparison of pi-rads version 2 and 2.1 in transition zone lesions for detection of prostate cancer: preliminary experience. *Journal of Magnetic Resonance Imaging*.

[9] Stolk T. T., de Jong I. J., Kwee T. C. (2019). False positives in PIRADS (V2) 3,4, and 5 lesions: relationship with reader experience and zonal location. *Abdominal Radiology*.

[10] Mertan F. V., Greer M. D., Shih J. H. (2016). Prospective evaluation of the imaging reporting and data version 2 for prostate cancer detection. *The Journal of Urology*.

[11] Tamura C., Shinmoto H., Soga S. (2014). Diffusion kurtosis imaging study of cancer: preliminary findings. *Journal of Magnetic Resonance Imaging*.

[12] Blystad I., Warntjes J. B. M., Smedby O., Landtblom A. M., Lundberg P., Larsson E. M. (2012). Synthetic MRI of the brain in a clinical setting. *Acta Radiologica*.

The article "Magnetic Resonance Image Compilation Was Used in Conjunction with Prostate PI-RADS v2.1 Score Has Diagnostic Relevance for Benign and Malignant Prostate Lesions" was retracted in 2023. Reasons: unreliable results or conclusions; concerns about the data; concerns about the peer review; concerns about the citations.

[13] Cui Y., Han S., Liu M. (2020). Diagnosis and grading of prostate cancer by relaxation maps from synthetic MRI. *Magnetic Resonance Imaging*.

[14] Engstrom M., Warntjes J. B., Tisell A., Landtblom A. M., Lundberg P. (2014). Multi-parametric representation of voxel-based quantitative magnetic resonance imaging. *PLoS One*.

[15] Gibbs P., Liney G. P., Pickles M. D., Zelhof B., Rodrigues G., Turnbull L. W. (2009). Correlation of ADC and T2 measurements with cell density in prostate cancer at 3.0 Tesla. *Investigative Radiology*.

[16] Liu W., Turkbey B., Sénégas J. (2011). Accelerated T2 mapping for characterization of prostate cancer. *Magnetic Resonance in Medicine*.

[17] Langer D. L., van der Kwast T. H., Evans A. J. (2010). Prostate tissue composition and MR measurements: investigating the relationships between ADC, T2, K(trans),v(e), and corresponding histologic features. *Radiology*.

[18] Gibbs P., Tozer D. J., Liney G. P., Turnbull L. W. (2001). Comparison of quantitative T2 mapping and diffusion-weighted imaging in the normal and pathologic prostate. *Magnetic Resonance in Medicine*.

[19] Sabouri S., Fazli L., Chang S. D. (2017). MR measurement of luminal water in prostate gland: quantitative correlation between MRI and histology. *Journal of Magnetic Resonance Imaging*.

[20] Sabouri S., Chang S. D., Savdie R. (2017). Luminal water imaging: a new MR imaging T2 mapping technique for prostate cancer diagnosis. *Radiology*.

[21] Mai J., Abubrig M., Lehmann T. (2019). T2 mapping in prostate cancer. *Investigative Radiology*.

[22] Mitchell D. G., Burk D. L., Vinitski S., Rifkin M. D. (1987). The biophysical basis of tissue contrast in extracranial MR imaging. *American Journal of Roentgenology*.

[23] van Houdt P. J., Agarwal H. K., van Buuren L. D. (2018). Performance of a fast and high-resolution mufti-echo spin-echo sequence for prostate T2 mapping across multiple systems. *Magnetic Resonance in Medicine*.

